RETRACTED

# Long noncoding RNA NORAD is upregulated in epithelial ovarian cancer and its downregulation suppressed cancer cell functions by competing with miR‐155‐5p

**DOI:** 10.1002/cam4.2350

**Published:** 2019-06-28

**Authors:** Lingling Tong, Yu Ao, Hejia Zhang, Kun Wang, Yunyun Wang, Qingjie Ma

**Affiliations:** ^1^ Department of Obstetrics and Gynecology China‐Japan Union Hospital of Jilin University Changchun China; ^2^ Department of Pediatric Intensive Care Unit (PICU) The First Hospital of Jilin University Changchun China; ^3^ Department of Ultrasonography China‐Japan Union Hospital of Jilin University Changchun China; ^4^ Department of Anesthesiology China‐Japan Union Hospital of Jilin University Changchun China; ^5^ Department of Nuclear Medicine China‐Japan Union Hospital of Jilin University Changchun China

**Keywords:** epithelial ovarian cancer, hsa‐miR‐155‐5p, lncRNA, miRNA, NORAD

## Abstract

**Purpose:**

In the present study, we evaluated the expression and function of human long noncoding RNA (lncRNA) activated by DNA damage (NORAD) in human epithelial ovarian cancer (EOC).

**Methods:**

NORAD expression was evaluated by qRT‐PCR in EOC cell lines and in situ EOC clinical samples. Lentivirus‐mediated NORAD downregulation was conducted in OVCAR‐3 and ES‐2 cells, and its effect on cancer cell proliferation, bufalin chemoresistance, cell‐cycle transition in vitro, and xenotransplantation in vivo were examined, respectively. The likelihood of an lncRNA‐microRNA (miRNA) signaling pathway was examined by probing the possible downstream competing target of NORAD, hsa‐miR‐155‐5p. Moreover, hsa‐miR‐155‐5p was knocked down in NORAD‐downregulated EOC cells to functionally evaluate the correlation between NORAD and hsa‐miR‐155‐5p in EOC.

**Results:**

We found that NORAD was substantially upregulated in both EOC cell lines and human tumors. In OVCAR‐3 and ES‐2 cells, lentivirus‐mediated NORAD downregulation had significant anticancer effects, as it suppressed cell proliferation, decreased bufalin chemoresistance, arrested cell‐cycle transition, and inhibited xenograft growth. Also, hsa‐miR‐155‐5p was confirmed to be the competing target of NORAD in EOC, and its knockdown in OVCAR‐3 and ES‐2 cells reversed the NORAD downregulation‐induced anticancer functions.

**Conclusions:**

NORAD is upregulated in EOC. Inhibition of NORAD, possibly through endogenously competing against hsa‐miR‐155‐5p, can be a new tumor‐suppressing strategy in EOC.

## 1 INTRODUCTION

Epithelial ovarian cancer (EOC) is one of the most lethal forms of gynecologic malignancy in women of age 40 or older.^1^, ^2^, ^3^ As estimated in 2018, there are more than 22 000 new cases of EOC and more than 14 000 EOC‐related deaths in the United States every year.^3^, ^4^ In China, these numbers are almost doubled, as the latest national cancer survey showed that there are annually more than 50 000 new cases of EOC and more than 22 000 EOC‐related deaths.^5^ In recent decades, although significant inside information had been gained toward the genetic mechanisms of EOC pathology, there has not been much improvement on early diagnosis or effective treatments to benefit cancer patients.^3^, ^5^ Thus, EOC patients are often diagnosed at late stages and suffered from poor prognosis and low survival rates.^3^, ^5^, ^6^

Long noncoding RNAs (lncRNAs) are groups of nonprotein‐coding RNAs (ncRNAs) that normally have a transcript of more than 200 nucleotides in length. In the recent decade, lncRNAs have been identified to play important roles, at both transcriptional and posttranscriptional levels, in modulating gene expressions and regulating a variety of physiological processes in eukaryotic cells.^7^, ^8^, ^9^ In addition, in human cancers, strong evidence has demonstrated that lncRNAs may be aberrantly expressed, either directly in tumor tissues or alternatively in circulating systems of cancer patients, thus having profound implications in prognosis prediction or cancer progression regulation in human patients.^10^, ^11^, ^12^

Of many of the lncRNAs which were found to be correlated with human cancers, Noncoding RNA activated by DNA damage (NORAD), a lncRNA comprising an exon located on Chr20q11.23, was demonstrated to be dysregulated (upregulated in most cases) in various types of human carcinomas, such as pancreatic cancer, colorectal cancer, breast cancer, or esophageal squamous cell carcinoma.^13^, ^14^, ^15^ Specifically, a very recent study showed that NORAD upregulated and modulated cancer cell proliferation and invasion in one of the most common gynecologic cancers, cervical cancer.^16^ However, it is still unknown whether NORAD may be dysregulated in another common type of gynecologic cancers, EOC, or whether NORAD may be actively participating in the functional regulation of cancer development in EOC.

RETRACTED

MicroRNAs (miRNAs) are another group of ncRNAs. However, unlike lncRNAs, miRNAs encode a very short‐length transcript, normally consisting of 18‐22 nucleotides. Like lncRNAs, epigenetic regulation by miRNAs has been found in almost every aspect of biological processes in eukaryotic cells, with miRNAs often posttranscriptionally inducing gene silencing through their downstream signaling pathways.^17^, ^18^, ^19^ Evidence also demonstrated that epigenetic crosstalk between lncRNAs and miRNAs may also play functional roles in cells, as lncRNAs could endogenously compete against binding miRNAs to either induce or inhibit downstream signaling pathways.^20^, ^21^ Specifically, in an effort to characterize lncRNA‐associated competing endogenous RNA networks (LCeNETs) in ovarian cancer, researchers used 401 clinical samples to identify more than 1,200 miRNA‐mediated crosstalk between lncRNAs and mRNAs.^22^

Thus, in the present study, we firstly evaluated the expression profile and functional roles of lncRNA NORAD in human EOC. Then, we sought the possible lncRNA‐miRNA crosstalk between NORAD and its competing target, predominant mature form of human microRNA‐155, microRNA‐155‐5p (hsa‐miR‐155‐5p, as opposed to the non‐predominant mature form of miR‐155, hsa‐miR‐155‐3p) in EOC. The purpose of our study is to seek the clarity of epigenetic regulation of lncRNA NORAD in human EOC.

## 2 MATERIALS AND METHODS

### 2.1 EOC Cell lines and clinical samples

An immortal normal human ovarian epithelial cell line, HS832.Tc, and seven human EOC cell lines, SK‐OV‐3, CAOV‐3, CAOV‐4, OVCAR‐3, HEY‐T30, ES‐2, and SW/626 were all commercially obtained from American Type Culture Collection (ATCC, USA). All cells were maintained in 6‐well tissue‐culture plates (VWR, USA) containing RPMI‐1640 medium (Thermo Fisher Scientific, USA) supplemented with 10% fetal bovine serum (FBS, MilliporeSigma, Shanghai, China) and 100 U/mL Penicillin‐Streptomycin (Pen/Strep, Thermo Fisher Scientific, USA) in a 5% CO_2 _tissue culture chamber at 37°C.

From September 2014 to December 2018, in situ EOC clinical samples, including EOC tumor samples and paired adjacent non‐tumor samples (at least 3 cm away from the clear edge of tumor) were excised from 17 patients diagnosed with EOC at Jilin University First Hospital and China‐Japan Union Hospital in Jilin City, China. Right after excision, clinical samples were snap‐frozen in liquid nitrogen and stored at −70°C until further processing.

### 2.2 RNA extraction and quantitative RT‐PCR

RNA extraction and quantitative RT‐PCR (qRT‐PCR) were performed on EOC cells and clinical samples based on our previously published methods, but with slight modification.^23^ Briefly, total RNA was extracted using an iPrep™ Trizol™ Plus RNA Kit (Invitrogen, USA), and verified using a NanoDrop 2000c spectrophotometer (Thermo Fisher Scientific, USA) according to the manufacturers' recommendations. A High‐Capacity cDNA Reverse Transcription Kit (Applied Biosystems, USA) was conducted to convert RNA into cDNA products. An ABI Prism 7000 Sequence Detection System (Applied Biosystems, USA) was used to conduct qRT‐PCR according to the manufacturer' recommendations. Measurement on lncRNA NORAD was conducted using a customized TaqMan™ NORAD noncoding RNA Assay, along with a control‐template 18S rRNA Taqman assay. Measurement on hsa‐miR‐155‐5p (Cat. No. 477927_mir) was conducted using a TaqMan™ Advanced miRNA assays and TaqMan^TM^ Fast Advanced Master Mix (Applied Biosystems, USA). RNU44 was used as a control template. Relative expressions were calculated against control samples using the 2^(−ΔΔCt)^ method.

RETRACTED

### 2.3 Lentivirus production and NORAD downregulation in EOC cells

Short hairpin RNA (shRNA) sequences specifically targeting human NORAD (NORAD_I), and a nonspecific human lncRNA shRNA (NS_I) were both designed and packaged into lentiviral vectors by RiboBio Biotechnology (RiboBio Biotech, Guangzhou, China). Transfection of NORAD_I or NS_I into human HEK293T cells with lentiviral packaging vectors to yield high‐titer lentiviruses was also manufactured and verified by RiboBio Biotechnology. In two EOC cell lines, OVCAR‐3 and CAOV‐4 cells were transduced with NORAD_I or NS_I lentiviruses in the presence of polybrene (10 μg/mL, MilliporeSigma, Shanghai, China) at multiplicity of infection (MOI) of 2 for 72 hours. A selection procedure was then carried out for 5‐7 days using blasticidin (15 μg/mL, MilliporeSigma, Shanghai, China). After that, clear‐edge healthy multicell colonies were collected, re‐plated in 6‐well plates containing fresh culture medium without blasticidin, and allowed to proliferate for 3‐5 passages, followed by qRT‐PCR analysis to verify the downregulation efficacy of endogenous NORAD expression.

### 2.4 In vitro proliferation assay

The method to evaluate EOC cancer cell proliferation in vitro was described in our previous study.^23^ Briefly, OVCAR‐3 and ES‐2 cells were lifted off from 6‐well plates and equally plated in a 96‐well plate at a concentration of 5000 cells/well for 5 days. At each proliferating day, EOC cells were firstly treated with a CellTiter 96^®^ Aqueous One Solution Cell Proliferation Assay (Promega, USA), and then examined on a spectraMax M3 multi‐mode microplate reader (Molecular Devices, USA). The in vitro EOC cell proliferating rates were measured at 490 nm wavelength absorbance.

### 2.5 In vitro chemoresistance assay

The method to assess EOC cancer cell in vitro chemoresistance was described in our previous study.^23^ Briefly, OVCAR‐3 and ES‐2 cells were lifted off from 6‐well plates and equally plated in a 96‐well plate at a concentration of 5000 cells/well. Bufalin (Sigma Aldrich, USA) was added into tested wells at various concentrations of 0, 0.25, 1, 5, and 10 ng/mL for 48 hours. After that, EOC wells were treated with 20 µL of CellTiter 96^®^ AQueous One Solution Reagent (Promega, USA) and examined on a spectraMax M3 multi‐mode microplate reader (Molecular Devices, USA). The relative percentages of healthy EOC cells were calculated by normalizing the absorbance recordings at 490 nm of all tested wells to the absorbance recordings of wells incubated with 0 ng/mL bufalin.

RETRACTED

### 2.6 In vitro cell‐cycle assay

The method to assess EOC cancer cell in vitro cell‐cycle stages was described in a previous study.^24^ Briefly, OVCAR‐3 and ES‐2 cells were quickly fixed and treated with propidium iodide (MilliporeSigma, Shanghai, China) for 1 hour at 37°C. Cell‐cycle stages, G0/G1, S, or M/G2, were determined using a FACSAria flow cytometer (BD Biosciences, USA) according to the manufacturer's instructions.

### 2.7 In vivo xenograft assay

The method to assess EOC cancer cell in vivo xenograft growth was described in our previous study.^23^ Briefly, 30 adult female athymic nude mice (6‐week‐old) were purchased from the Shanghai Slac Laboratory Animal Company (SLAC, Shanghai, China). Lentiviral‐transduced OVCAR‐3 cells were injected (1 × 10^6^ cells/injection) into the subcutaneous lower flanks of those mice, with 15 mice injected with NS_I‐transduced OVCAR‐3 cells and 15 mice injected with NORAD_I‐transduced OVCAR‐3 cells. The in vivo xenograft assay was conducted for 5 weeks. Tumor volumes (v, mm^3^) were estimated weekly using the formula, v = L*W*W/2, with L representing lengths (mm) and W representing widths (mm). Five weeks later, mice were sacrificed and OVCAR‐3 xenografts were excised for visual examination.

### 2.8 Dual‐luciferase reporter assay

A synthetic human mature hsa‐miR‐155‐5p mimics (miR155‐m) and a nonspecific human miRNA mimics (miRNS‐m) were purchased from RiboBio Biotechnology (RiboBio Biotech, Guangzhou, China). The 3′‐UTR of human NORAD gene, including two fragments of putative hsa‐miR‐155‐5p binding sites, was amplified by PCR and sub‐cloned into a pGL3 luciferase reporter plasmid to generate a wild‐type NORAD luciferase‐reporter vector, WT(NRD). In addition, the two DNA fragments of putative hsa‐miR‐155‐5p binding sites were individually point‐mutated and sub‐cloned into pGL3 to generate mutant NORAD luciferase‐reporter vectors, MU(NRD)_1 and MU(NRD)_2. Alternatively, two putative hsa‐miR‐155‐5p binding sites were both point‐mutated. And that, mutant NORAD 3′‐UTR sequence was sub‐cloned into pGL3 to generate third mutant NORAD luciferase‐reporter vector, MU(NRD)_1_2. Then, in the culture of immortal human embryonic kidney cells 293T (HEK293T), cells were cotransfected with miR155‐m or miRNS‐m, along with luciferase‐reporter vectors of WT(NRD), MU(NRD)_1, MU(NRD)_2, or MU(NRD)_1_2. A dual‐luciferase reporter assay was then carried out according to the method in our previous publication.^23^ Relative luciferase activities were normalized to the values in HEK293T cells cotransfected with miRNS‐m and WT(NRD).

RETRACTED

### 2.9 Hsa‐miR‐155‐5p downregulation in EOC cells

A synthetic human mature hsa‐miR‐155‐5p inhibitor (miR155_I) and a nonspecific human miRNA inhibitor (miRNC_I) were purchased from RiboBio Biotechnology (RiboBio Biotech, Guangzhou, China). In OVCAR‐3 and ES‐2 cells stably transduced with NORAD_I, we double transfected them with miR155_I or miRNC_I using Lipofectamine 3000 transfection reagent (MilliporeSigma, Shanghai, China) for 48 hours, followed by qRT‐PCR analysis to verify the downregulation efficacy on endogenous hsa‐miR‐155‐5p expression.

### 2.10 Statistical analysis

All experiments were independently performed in at least three biological repeats. The averaged values were shown as means ± SEM Statistical analysis was performed using a Windows‐based SPSS software (SPSS, version 13.0, USA) and measured by one‐way ANOVA with Tukey's post hoc test. *P*‐values < 0.05 were considered as significant difference.

## 3 RESULTS

### 3.1 NORAD is upregulated in EOC cells and human EOC tumors

We evaluated NORAD expression in immortal EOC cell lines, including SK‐OV‐3, CAOV‐3, CAOV‐4, OVCAR‐3, HEY‐T30, ES‐2, and SW/626 cells. The analysis of qRT‐PCR showed that, in all tested EOC cells, NORAD expressions were significantly higher than NORAD expression in an immortal normal human ovarian epithelial cell line, HS832.Tc (Figure 1A, * *P* < 0.05). Also, we evaluated NORAD expression in in situ human EOC tumors. In 17 patients diagnosed with EOC, NORAD was compared between tumor tissues and paired adjacent non‐tumor samples. The analysis of qRT‐PCR demonstrated that, in 15 of 17 cases, NORAD was significantly upregulated in EOC tumor tissues than non‐tumor tissues (Figure 1B, *P < 0.05). In the other two cases, NORAD expressions were seemingly higher in EOC tumor tissues than paired non‐tumor tissues, but without statistical significance (Figure 1B, ∆*P* > 0.05).

**Figure 1:** Expression of lncRNA NORAD in EOC. A, LncRNA NORAD expressions were evaluated by qRT‐PCR in in vitro EOC cell lines, SK‐OV‐3, CAOV‐3, CAOV‐4, OVCAR‐3, HEY‐T30, ES‐2, and SW/626 cells, and compared to endogenous NORAD expression in an immortal normal human ovarian epithelial cell line, HS832.Tc (*P < 0.05). B, LncRNA NORAD expressions were also evaluated by qRT‐PCR between 17 pairs of in situ EOC human tumors and their adjacent non‐tumor epithelial tissues (*P < 0.05; ∆*P* > 0.05).

### 3.2 NORAD downregulation exhibited anticancer effects on EOC in vitro proliferation and chemoresistance

Lentiviral transduction was applied on OVCAR‐3 and ES‐2 cells to downregulate NORAD expression. After transduction was stabilized, analysis of qRT‐PCR showed cells transduced with NORAD_I lentivirus had significantly lower NORAD expressions than cells transduced with NS_I lentivirus (Figure 2A, *P < 0.05).

RETRACTED

**Figure 2:** NORAD downregulation inhibited proliferation and chemoresistance of EOC cells. A, Two EOC cell lines, OVCAR‐3 and ES‐2 cells, were transduced with lentiviruses of NORAD_I (NORAD‐specific shRNA) or NS_I (nonspecific control). After transduction was stable in EOC cells, their endogenous NORAD expressions were compared by qRT‐OCR (*P < 0.05). B, For OVCAR‐3 and ES‐2 cells transduced with lentiviruses of NORAD_I or NS_I, they were re‐plated in 96‐well plates, to be evaluated by an in vitro proliferation assay for 5 d. Each day, absorbance at 490‐nm wavelength was recorded, and compared between NIS_I‐ and NORAD_I‐transduced EOC cells (*P < 0.05). C, Lentiviral‐transduced OVCAR‐3 and ES‐2 cells were also treated with bufalin at concentrations (ng/mL) of 0, 0.25, 1, 5, and 10 for 48 h. Relative percentages of healthy cells, representing cancer cell bufalin chemoresistance, were compared between NS_I‐ and NORAD_I‐transduced EOC cells (*P < 0.05)

Then, lentiviral‐transduced OVCAR‐3 and ES‐2 cells were evaluated by an in vitro proliferation assay. It showed that, cancer cell proliferating rates were significantly slower in OVCAR‐3 and ES‐2 cells transduced with NORAD_I, as compared to those transduced with NS_I (Figure 2B, *P < 0.05).

Also, lentiviral‐transduced OVCAR‐3 and ES‐2 cells were evaluated by an in vitro chemoresistance assay, with the treatment of bufalin at various concentrations (0‐10 ng/mL) for 48 hours. The result demonstrated that, bufalin chemoresistance was significantly reduced in OVCAR‐3 and ES‐2 cells transduced with NORAD_I, as compared to those transduced with NS_I (Figure 2C, *P < 0.05).

Thus, our data suggested that NORAD downregulation had significant anticancer effects on EOC proliferation and bufalin chemoresistance.

### 3.3 NORAD downregulation exhibited anticancer effects on EOC in vitro cell‐cycle transition and in vivo xenograft growth

We then evaluated the effect of NORAD downregulation on EOC cell‐cycle transition in vitro. The DNA contents of lentiviral‐transduced OVCAR‐3 and ES‐2 cells were evaluated using a flow‐cytometry cell‐cycle assay. It showed that, in both OVCAR‐3 and ES‐2 cells, G0/G1 stages were significantly extended and S stages significantly shortened in cells transduced with NORAD_I than those transduced with NS_I (Figure 3A, *P < 0.05).

**Figure 3:** NORAD downregulation arrested EOC cell‐cycle and suppressed EOC in vivo growth. A, For OVCAR‐3 and ES‐2 cells transduced with lentiviruses of NORAD_I or NS_I, they were cultured until>~80% confluency, quickly fixed and evaluated by flow cytometry. The percentages of EOC cells at different cell‐cycle stages, G0/G1, S, and M/G2, were then compared between NS_I‐ and NORAD_I‐transduced EOC cells (*P < 0.05). B, OVCAR‐3 cells, transduced by either NS_I or NORAD_I, were inoculated into subcutaneous flanks of 30 athymic nude mice (15 mice received NS_I‐transduced cells and the other 15 mice received NORAD_I‐transduced cells) for 5 wk. The in vivo tumor volumes were compared weekly between NS_I‐ and NORAD_I‐transduced xenografts (*P < 0.05). C, Post xenograft assay, NS_I‐ and NORAD_I‐transduced OVCAR‐3 tumors were excised from host mice and compared.

RETRACTED

In addition, we evaluated the effect of NORAD downregulation on in vivo growth of EOC xenograft. Lentiviral‐transduced OVCAR‐3 cells were subcutaneously injected into a mouse xenograft model for 5 weeks, with their tumor volumes compared weekly. The comparison showed that, in vivo subcutaneous tumor volumes were dramatically decreased in OVCAR‐3 xenografts transduced with NORAD_I than those transduced with NS_I (Figure 3B, *P < 0.05). Post xenograft model, OVCAR‐3 tumors were excised and compared. It demonstrated that NORAD_I‐transduced xenografts were markedly smaller than NS_I transduced xenografts (Figure 3C).

Thus, our data further demonstrated that NORAD downregulation had significant anticancer effects on EOC cell‐cycle transition and xenotransplantation.

### 3.4 NORAD is competing with hsa‐miR‐155‐5p in EOC

By searching lncRNA downstream target database of StarBase v2.0,^25^, ^26^ it was revealed that human microRNA hsa‐miR‐155‐5p could be possibly bound by two DNA fragments on NORAD 3′‐UTR, thus making hsa‐miR‐155‐5p a possible downstream competing candidate of NORAD (Figure 4A,B). Based on these information, we constructed four luciferase‐reporter vectors, WT(NRD), MU(NRD)_1, MU(NRD)_2, and MU(NRD)_1_2, and cotransfected them with miR155‐m or miRNS‐m in HEK293T cells. Forty‐eight hours later, a dual‐luciferase reporter assay demonstrated that, in cells transfected with WT(NRD), MU(NRD)_1, or MU(NRD)_2, cotransfection with miRNS‐m or miR155‐m yielded a significant difference in relative luciferase activities (Figure 4C, *P < 0.05). However, in cells transfected with MU(NRD)_1_2, cotransfection with miRNS‐m or miR155‐m did not show any difference in relative luciferase activities (Figure 4C, ∆*P* > 0.05). Therefore, the result of our dual‐luciferase activity assay confirmed that NORAD could directly bind hsa‐miR‐155‐5p.

**Figure 4:** NORAD is negatively correlated with hsa‐miR‐155‐5p in EOC. (A & B) Transcript sequences are shown for two wild‐type (WT) NORAD 3′‐UTR fragments (A, WT(NRD) fragment 1; B, WT(NRD) fragment 2) with putative binding sites of hsa‐miR‐155‐5p. In addition, two binding sites were individually mutated (A, MU(NRD)_1; B, MU(NRD)_2). (C) HEK293T cells were cotransfected with miR155‐m or miRNS‐m, along with luciferase‐reporter vectors containing wild‐type or mutant NORAD 3′‐UTR (WT(NRD), MU(NRD)_1, MU(NRD)_2, MU(NRD)_1_2). A dual‐luciferase reporter assay was conducted for 48 h. For HEK293T cells transfected with different luciferase‐reporter vectors, relative luciferase activities were compared between miRNS‐m and miR155‐m cotransfected cells (*P < 0.05, ∆*P* > 0.05). (D) For OVCAR‐3 and ES‐2 cells transduced with lentiviruses of NORAD_I or NS_I, their endogenous hsa‐miR‐155‐5p expressions were compared by qRT‐PCR (*P < 0.05). (E) Coexpression correlation was shown for 376 clinical samples of ovarian serous cystadenocarcinoma (Cited from: Pan‐Cancer database, http://starbase.sysu.edu.cn/panMirCoExp.php).

RETRACTED

In addition, in lentiviral‐transfected OVCAR‐3 and ES‐2 cells, qRT‐PCR analysis demonstrated that miR‐155‐5p was reversely upregulated by NORAD downregulation (Figure 4D, *P < 0.05).

Moreover, we examined the coexpression pattern of NORAD and hsa‐miR‐155‐5p in ovarian serous cystadenocarcinoma using Pan‐Cancer database (http://starbase.sysu.edu.cn/panMirCoExp.php), and found out that NORAD and hsa‐miR‐155‐5p expressions were statistically correlated (Figure 4E).

Thus, all those data strongly support the hypothesis that NORAD is competing with hsa‐miR‐155‐5p in EOC.

### 3.5 Hsa‐miR‐155‐5p inhibition reversed the anticancer functions of NORAD downregulation in EOC cells

Finally, we hypothesized that hsa‐miR‐155‐5p is functionally involved in the anticancer regulations of NORAD downregulation in EOC. In OVCAR‐3 and ES‐2 cells with stable NORAD downregulation, or those transduced with NORAD_I, we double‐infected them with a synthetic hsa‐miR‐155‐5p inhibitor (miR155‐I), or a nonspecific miRNA inhibitor (miRNC_I). Then, analysis of qRT‐PCR showed that transfection of miR155‐I significantly inhibited (or downregulated) hsa‐miR‐155‐5p expression in OVCAR‐3 and ES‐2 cells pre‐transduced with NORAD_I (Figure 5A, *P < 0.05).

**Figure 5:** Hsa‐miR‐155‐5p inhibition had an opposite function as NORAD downregulation in EOC cells. A, For OVCAR‐3 and ES‐2 cells transduced with lentiviruses of NORAD_I, they were double transfected with either miR155‐I or miRNS‐I. After that, qRT‐PCR was applied to compare their endogenous hsa‐miR‐155‐5p expressions (*P < 0.05). B, For double‐infected OVCAR‐3 and ES‐2 cells, they were re‐plated in 96‐well plates, to be evaluated by an in vitro proliferation assay for 5 d. Each day, absorbance at 490‐nm wavelength was recorded, and compared between EOC cells infected with NORAD _I and miR155_I and cells infected with NORAD _I and miRNC_I (*P < 0.05). C, Double‐infected OVCAR‐3 and ES‐2 cells were also treated with bufalin at concentrations (ng/ml) of 0, 0.25, 1, 5, and 10 for 48 h. Relative percentages of healthy cells, representing cancer cell bufalin chemoresistance, were compared between EOC cells infected with NORAD _I and miR155_I and cells infected with NORAD _I and miRNC_I (*P < 0.05). D, For double‐infected OVCAR‐3 and ES‐2 cells, they were cultured until>~80% confluency, quickly fixed and evaluated by flow cytometry. The percentage of EOC cells at different cell‐cycle stages, G0/G1, S, and M/G2, were then compared between EOC cells infected with NORAD _I and miR155_I and cells infected with NORAD _I and miRNC_I (*P < 0.05).

RETRACTED

Then double‐infected OVCAR‐3 and ES‐2 cells were evaluated by the in vitro proliferation assay. It showed that, cancer cell proliferating rates were significantly prompted in OVCAR‐3 and ES‐2 cells double‐infected with NORAD_I and miR155_I, as compared to those double‐infected with NORAD_I and miRNC_I (Figure 5B, *P < 0.05).

Also, double‐infected OVCAR‐3 and ES‐2 cells were evaluated by the in vitro chemoresistance assay, also with the treatment of bufalin at various concentrations (0‐10 ng/mL) for 48 hours. The result demonstrated that bufalin chemoresistance was drastically reduced for OVCAR‐3 and ES‐2 cells double‐infected with NORAD_I and miR155_I, as compared to those double‐infected with NORAD_I and miRNC_I (Figure 5C, *P < 0.05).

Furthermore, we evaluated DNA contents of double‐infected OVCAR‐3 and ES‐2 cells using an in vitro flow‐cytometry cell‐cycle assay. The result showed that, G0/G1 stages were significantly shortened and S stages significantly extended in OVCAR‐3 and ES‐2 cells double‐infected with NORAD_I and miR155_I, as compared to those double‐infected with NORAD_I and miRNC_I (Figure 5D, * *P* < 0.05).

Thus, our data clearly indicated that hsa‐miR‐155‐5p is a functional competing target of NORAD in regulating EOC cells.

## 4 DISCUSSION

Mounting evidence has demonstrated that epigenetic regulation of lncRNAs plays important roles in human cancer progression, and may hold the key to developing novel molecular target for cancer treatment.^10^, ^11^, ^12^ In the present study, we presented new data, showing lncRNA NORAD is upregulated in human EOC and inhibiting NORAD could yield tumor‐suppressing functions in EOC cells through endogenously competition against hsa‐miR‐155‐5p.

RETRACTED

As the first step of our study, we used a quantitative method to reveal that NORAD was upregulated in both immortal EOC cell lines and in situ EOC human tumors. In seven evaluated EOC cell lines, we found NORAD expressions were upregulated in all cell lines. In addition, NORAD upregulation was discovered in 15 of 17 cases of EOC tumors. In the other two cases, NORAD did show increased expression patterns in tumor tissues than adjacent non‐tumor tissues, though the differences were not significant. In several previously published studies, NORAD was also found to be upregulated (or overexpressed) in other human carcinomas, such as pancreatic cancer,^14^ breast cancer,^27^ or colorectal cancer.^15^ By combining these evidences, it seems like NORAD is very likely to be aberrantly upregulated in not one, but many types of human cancers. However, it is worth noting that our analysis on in situ clinical tissues may indicate heterogeneous expression pattern of NORAD in human EOC, as NORAD was not significantly upregulated in EOC tumors in two cancer patients. Thus, future investigation is required to further elucidate the correlation between NORAD expression and clinicopathological parameters of EOC patients.

Next in our study, we adapted lentiviral transduction to successfully downregulate NORAD in OVCAR‐3 and ES‐2 cells. Then, through several biochemical assays, we provided strong evidence showing NORAD inhibition had significant anticancer effects on both in vitro and in vivo cancer cell functions. These findings are consistent with the upregulated expression pattern of NORAD in EOC cells and suggest an oncogenic role of NORAD in EOC. Then, it is perhaps not surprising to see similar functional roles of NORAD in other types of human cancers, as downregulating NORAD also yielded significant inhibitory effects on proliferation and migration in both pancreatic cancer and breast cancer cells.^15^, ^27^ However, the present study is the first report demonstrating the mechanistic role of NORAD in human EOC cells.

The most significant findings of our study might be the discovery of the endogenous competing mechanism between NORAD and hsa‐miR‐155‐5p. To support this finding, it was demonstrated that hsa‐miR‐155‐5p (hsa‐miR‐155) was found to be a tumor suppressor in ovarian cancer‐initiating cells,^28^ and the inverse coexpression correlation between NORAD and hsa‐miR‐155‐5p was revealed through Pan‐Cancer Study using nearly 400 clinical samples of ovarian serous cystadenocarcinoma (Figure 4E, http://starbase.sysu.edu.cn/panMirCoExp.php). In addition, in lentiviral‐transduced EOC cells, we found that hsa‐miR‐155‐5p was inversely upregulated by NORAD downregulation (Figure 4D). Furthermore, while we conducted double‐infection to downregulate hsa‐miR‐155‐5p in NORAD‐downregulated EOC cells, it was demonstrated that NORAD downregulation‐induced tumor‐suppressing effects on cancer cell proliferation, chemoresistance, and cell‐cycle transition were all significantly and functionally reversed. Thus, those results all support the notion that NORAD is endogenously competing against hsa‐miR‐155‐5p in human EOC.

RETRACTED

It is intriguing to note that, our data of dual‐luciferase activity assay (Figure 4C) suggest that it may require two binding sites to be active for NORAD to effectively modulate hsa‐miR‐155‐5p and its downstream signaling pathways. A future quantitative study, possibly comparing the cope numbers of NORAD and hsa‐miR‐155‐5p transcripts in human patients may provide more details on how exactly NORAD may bind hsa‐miR‐155‐5p and compete against its downstream signaling pathways.

## CONFLICT OF INTEREST

None to be declared.
